RETRACTED

# Improvement of the Accuracy in the Identification of Coronary Artery Disease Combining Heart Sound Features

**DOI:** 10.1155/2022/3058835

**Published:** 2022-02-23

**Authors:** Haixia Li, Guojun Zhang, Guicheng Shao, Aizhen Wang, Yarong Gu, Zhumei Tian, Qiong Zhang, Pengcheng Shi

**Affiliations:** ^1^Department of Electronics, Xinzhou Teachers University, Xinzhou, China; ^2^State Key Laboratory of Dynamic Testing Technology, North University of China, Taiyuan, China

## Abstract

Most researchers use features of diastolic murmurs to identify coronary artery disease. However, the diastolic murmurs of coronary artery disease are usually very weak and are easily contaminated by noise and valvular murmurs. Therefore, the diagnostic accuracy of coronary artery disease when only using diastolic murmurs is not well. An algorithm for improving the accuracy in the identification of coronary artery disease by combining the features of the first heart sound and diastolic murmurs was proposed. Firstly, a first heart sound feature extraction algorithm was used to identify coronary artery disease from noncoronary artery disease. Secondly, the Empirical Wavelet Transform algorithm was used to decompose the diastolic heart sound into three modes, and the spectral energy of each mode was calculated to distinguish coronary artery disease from noncoronary artery disease. Then, the features of the fist heart sound, the second diastolic spectral energy, and the parameter P3, which was used to discriminate the diastolic murmurs in coronary artery disease and in valvular disease, were combined together to improve the diagnostic accuracy of coronary artery disease. The comparison experiment results show that the accuracy of the proposed algorithm is superior to some state-of-the-art methods when they are used to diagnose coronary artery disease.

## 1. Introduction

Coronary artery disease (CAD), identified by the World Health Organization as the “number one killer”, kills about 17.3 million people each year globally, and it is expected to increase to 23.6 million by 2030 [1]. According to “China's Health and Family Planning Statistical Yearbook (2018)” [2], the current situation of prevention and treatment of CAD is not optimistic. Its mortality rate continues to rise year by year (as shown in Figure 1), and there has always been a “three low” situation—low diagnosis rate, low treatment rate, and low control rate. One-third of the patients with CAD encountered myocardial infarction, heart failure, or other serious events when they first presented clinical symptoms of CAD and died without the opportunity to receive targeted treatment [3]. The reason of this is that the commonly used CAD detection methods are usually expensive, invasive, inconvenient, and unable to realize the accurate early detection of CAD [4–9]. The literature has shown that when the coronary arteries are blocked by 30%, there is a specific response to heart sounds [10]. Therefore, the detection of heart sounds is expected to realize the early noninvasive diagnosis of CAD. In recent years, with the successful development of electronic stethoscopes and the digital signal processing technology, the extraction of heart sound characteristic parameters to assist the diagnosis of various cardiovascular diseases has once again become a research hotspot globally [11–13].

RETRACTED

### 1.1. Related Works and Motivation

The diagnostic methods of CAD are classified into two categories: invasive diagnosis and noninvasive diagnosis. Noninvasive diagnostic techniques for CAD are generally on the bases of the electrical activity and pumping activity of heart, such as ECG (electrocardiogram), dynamic ECG, echocardiography, NMR (nuclear magnetic resonance), CT (computer tomography), and PET-CT (positron emission computed tomography). The invasive CAD detection mainly refers to coronary arteriography.

Electrocardiogram (ECG) is the earliest, most commonly used, and most basic diagnostic method for CAD. But not all patients with CAD can be diagnosed by ECG. If the degree of coronary artery stenosis is light, the heart can also maintain the need for myocardial blood supply under normal circumstances. Then, ECG is normal. Therefore, it is difficult to achieve the early diagnosis of CAD using ECG [6].

An ECG load test is for patients with suspected CAD but normal ECG. After increasing the patients' activity and the burden of heart, ECG may become abnormal and the symptoms of myocardial ischemia may be identified. The ECG load test plays a certain role in improving the diagnostic rate of CAD only using ECG. However, the load test is not suitable for some old and weak people with limited mobility [6].

Echocardiography can show the size of each chamber of the heart, the thickness of interventricular septum and ventricular wall, and the active state of each valve. For a CAD patient, echocardiography can reflect the change of its heart structure and the decrease of heart function. However, not all patients with CAD have these changes. If the degree of coronary blockage is light, echocardiography can be normal [7].

The current isotopic myocardial scanning has a certain value in the diagnosis of CAD. In the quiet state, the amount of radioisotopes entering the ischemic area due to compensatory action was similar to that entering the normal myocardium, and the scan showed a uniform distribution of radioactivity. When the myocardial oxygen consumption increases significantly after exercise, the coronary artery blood flow also increases correspondingly. However, due to coronary artery stenosis, blood flow cannot be increased correspondingly in ischemic areas. Therefore, the amount of radioisotopes entering the normal myocardium is significantly different from the amount entering the diseased myocardium, which can be used to diagnose CAD. Because coronary perfusion has a strong reserve capacity, it is not meaningful when coronary stenosis is relatively mild.

RETRACTED

Modern medical imaging technologies, such as NMR, CT, and PET, have powerful functions and can intuitively show the pathological state of the heart [8, 9]. The main problem is the high cost of such method, which cannot be accepted unless the patient has obvious symptom of heart disease. And this kind of equipment is complex to use and difficult to maintain.

Coronary angiography is currently the “gold standard” for the diagnosis of CAD, which can determine whether the coronary artery has stenosis and the location and degree of the stenosis. However, coronary angiography is an invasive detection method with certain risks, serious complications, and even death. The mortality rate of the relevant data is around 0.1%. Moreover, the process is complicated and expensive, which makes it unsuitable for large-scale detection of CAD [5, 10].

Previous studies have shown that, driven by blood pressure, blood flowing through the stenosis of coronary arteries will consume more energy. After blood flowing through the stenosis, separation between the flow layers will occur at the expansion of the outlet, and further vortices will form. Therefore, high-frequency murmurs will occur in diastolic heart sound when stenosis occurs due to coronary artery occlusion [14–17]. The findings show that CAD is associated with increased diastolic energy above 200-300 Hz [7–9]. Multiple methods have been applied for identification of the resonance related components. In 1992, Akay adopted the adaptive filtering method to eliminate the background noise of cardiac diastolic signals, established the ARMA and AR models of cardiac diastolic signals, and used the power spectrum and pole models as diagnostic parameters and obtained many valuable results. Dragomir et al. used fast Fourier transform (FFT) to analyze the diastolic spectra of coronary artery disease patients before and after stenting [10]. The CAD signature was evaluated by estimating power ratios of the total power above 150 Hz over the total power below 150 Hz of the FFT of the acoustic signal. Makaryus et al. used Wavelet analysis to extract the difference between CAD and normal subjects in diastolic heart sounds [12]. Winther et al. used the eigenvector method to study the diastolic heart sound of coronary artery stenosis before and after angioplasty and showed that the diastolic murmurs were equivalent to a narrowband signal with high frequency, which were associated with coronary artery stenosis [17]. Akay et al. applied EMD (empirical mode decomposition) algorithm and Hilbert Transformation to analyze the diastolic heart sound of CAD and found that the average instantaneous frequency of diastolic heart sounds in patients with CAD is higher than that of normal subject [18]. Schmidt et al. used a CAD-score which was produced from nine different types of features from five overlapping diastolic frequency bands to identify CAD [15]. Wavelet analysis [19], fast tracking filters [20], and parametric models [21] were also used to identify the diastolic murmurs associated with CAD.

RETRACTED

### 1.2. Objective and Key Contributions

As a matter of fact, diastolic high-frequency murmurs can be caused by other valvular diseases either [4]. Moreover, diastolic high-frequency murmurs are very weak, which can be filtered as noise easily. Therefore, the accuracy in the diagnosis of CAD using heart sound analysis can be further improved.

Reference [4], one of our previous studies, has proved that valvular disease could cause diastolic murmurs and proposed a method to distinguish the diastolic murmurs between in CAD and in valvular disease. P3, the ratio of spectral energy greater than 250 Hz and spectral energy less than 250 Hz in the third diastolic modal spectrum, can be used as the feature parameter to directly distinguish diastolic murmurs in CAD and in valvular disease. Reference [24], another one of our previous studies, proposed a method to detect and classify the abnormities of first heart sound (S1). In that paper, S1s were divided into three categories: normal S1, S1 with abnormal split, and S1 with abnormal amplitude. The heart sounds in our previous studies come from Michigan Heart Sounds Database, and our own database collected by ourselves made a MEMS electronic stethoscope [23]

Therefore, the key contributions of this paper are

1. an investigation of the effectiveness of the proposed method in reference [20] for discriminating the S1 of CAD and non-CAD since the common characteristics of clinical auscultation of CAD are weak heart contractions and weakened first heart sound (S1) [17]
2. an investigation of the effectiveness of the Empirical Wavelet Transform (EWT) for discriminating the second diastolic spectral energy *e*(2) of CAD and non-CAD, in which *e*(2) is the spectral energy corresponding to the 150~500 Hz of diastolic heart sounds
3. a pioneer combining features of S1 and *e*(2) and P3 to distinguish CAD from non-CAD in order to improve the accuracy in diagnosis of CAD based on feature extraction of heart sounds

Until now, no one has studied the characteristic features of S1 in CAD. The proposed method which combines features of S1 and *e*(2) and P3 to distinguish CAD from non-CAD is for the first time. Through comparative studies, the effectiveness of the proposed method in improving the accuracy of the identification of CAD and non-CAD has been proved.

RETRACTED

This paper is organized as follows: Section 2 describes the details of the proposed method.  Section 3 presents the processing results of each subalgorithm when the proposed method was applied to deal with different heart sounds.  Section 4 is the conclusion of this study.

## 2. Methodology

The proposed method consists of three subalgorithms: feature extraction of first heart sound of CAD, feature extraction of P3, and feature extraction of diastolic murmurs using EWT. The literature [4] focuses on the calculation of P3, which was used to distinguish diastolic murmurs between in CAD and in valvular disease. This section focuses on the subalgorithm of S1 feature extraction applied in distinguishing CAD from non-CAD and subalgorithm of feature extraction of diastolic murmurs in CAD.  Figure 2 shows the details and steps of the proposed method.

### 2.1. Feature Extraction of First Heart Sound of CAD

Clinical auscultations of CAD are weak heart contractions and weakened first heart sound (S1). Using the proposed method in Reference [24], the characteristics of CAD's S1s are comparatively studied. It is well known that S1 mainly consists of two main frequency components, namely, M1—the frequency component produced by mitral valve closure and T1—the frequency component produced by tricuspid valve closure [22]. By analyzing the changes of instantaneous frequency (IF) of M1 and T1, abnormalities of S1 can be detected and classified.

At first, after extracting the envelop of heart sound by the Shannon Energy, S1s are extracted by algorithms of double threshold segmentation and localization. Then, Empirical Wavelet Transform (EWT) is applied to divide the spectrum of S1. The EWT algorithm divides the Fourier spectrum of a signal to construct some wavelet filter banks and extracts the AM-FM components of the signal with tight support spectrum through orthogonal Empirical Wavelet Transform (EWT). In order to find the right instantaneous frequency (IF) of M1 and T1 accurately and quickly, the peak values in the S1s' spectrum are sorted firstly. Then, the first two maximum values located with a distance greater than 20 Hz are selected. The nearest minimum values on both sides of the selected maximum values are used as the boundary points to divide the spectrum of S1.

RETRACTED

Secondly, S1s are decomposed into five modes according to the segmentation of the spectrum. Only the second mode and the fourth mode signals are single-frequency components. The other modal components have no practical significance. The second and fourth modes correspond exactly to the maximum subsignals of M1 and T1.

Thirdly, the instantaneous frequency (IF) of each modal signal is calculated through Hilbert Transform, and the *k*-means algorithm is used to carry out clustering analysis of the IF of the five modes. The IF of second mode and the fourth mode can form continuous curve after Hilbert Transform and *k*-means clustering analysis. The values of time, frequency, and amplitude corresponding to the IF with the maximum amplitude in M1 and T1 can be easily found.

Hilbert Huang Transform (HHT) is defined as (1), (2), (3), (4), (5) and (6)

(1) $$\begin{array}{c} \hat{x}\left(t\right)=H\left[x\left(t\right)\right]=\frac{1}{\pi }\int_{-\infty }^{+\infty }\frac{x\left(\tau \right)}{t-\tau }d\tau =x\left(t\right)*h\left(t\right), \end{array}$$

where *h*(*t*) = 1/*πt*, ∗ means convolution operation. *x*(*t*) is each filter's output and $\hat{x}\left(\text{t}\right)$ is the result of Hilbert Transform. An analytical signal is constructed with $\hat{x}\left(t\right)$ as the imaginary part, denoted as

(2) $$\begin{array}{c} z\left(t\right)=x\left(t\right)+j\hat{x}\left(t\right)=\alpha \left(t\right)e^{j\theta \left(t\right)}, \end{array}$$

(3) $$\begin{array}{c} \alpha \left(t\right)=\sqrt{x{\left(t\right)}^{2}+\hat{x}{\left(t\right)}^{2}}, \end{array}$$

(4) $$\begin{array}{c} \theta \left(t\right)=\arctan\frac{\hat{x}\left(t\right)}{x\left(t\right)}. \end{array}$$

This analytical signal's instantaneous frequency can be expressed as

(5) $$\begin{array}{c} f\left(t\right)=\frac{1}{2\pi }\frac{d\theta \left(t\right)}{dt}. \end{array}$$

After all the modes are evaluated using Hilbert Transform, the analytical signal can be expressed as

(6) zt=Re∑i=1nαitejθt=Re∑i=1naiej∫witdt.

Equation (6) reveals how the signal's IF varies with time and its amplitude.

The values of the amplitude, frequency, and time interval of the IF of different S1's M1 and T1 are different and have their own characteristics. The comparative study results will be presented in the next section.

### 2.2. Feature Extraction of Diastolic Murmurs Using EWT

Pathological heart sounds often contain all kinds of systolic and diastolic murmurs or S3 and S4 both in CAD and in valvular heart disease, which will make the segmentation of diastolic heart sound become difficult and then greatly affect the accuracy of CAD's identification based on the feature extraction of diastolic murmurs. The wavelet threshold denoising algorithm is used to denoise the heart sound signal firstly [4].

RETRACTED

The noise type of heart sound data collected by MEMS electronic stethoscope is simple, and the wavelet threshold denoising algorithm is used to denoise heart sound data. Sym3 wavelet basis and three-layer decomposition can be uniformly adopted. The threshold function is uniformly set as [24]

(7) $$\begin{array}{c} \beta_{j}=\sigma_{j}^{\text{Noise}}\sqrt{2\log\left(N_{j}\right)}. \end{array}$$

*N*_*j*_ is the length of the signal at the decomposition scale or layer *j*.  *σ*_*j*_^Noise^ is the noise variance of layer *j*; it can be calculated through formula (8) where *CD*_*j*_ is the detail component of wavelet decomposition in layer *j*.

(8) $$\begin{array}{c} \sigma_{j}^{\text{Noise}}=\frac{\text{median}\left(\left|CD_{j}\right|\right)}{0.6745}. \end{array}$$

Secondly, according to the different frequency distribution ranges of heart sounds and murmurs, the Empirical Wavelet Transform (EWT) is used to separate the murmurs and heart sounds, and then, the double threshold segmentation algorithm is used to extract the pure diastolic heart sounds, and finally, the original diastolic heart sounds with murmurs can be extracted according to the position of the pure diastolic heart sounds.

Thirdly, in order to extract the coronary blood flow with maximum diastolic murmur and clearly avoid acoustic interference of the valve cover, a fixed window function is used to extract diastolic heart sounds from each cardiac cycle: a period of 128 ms starting at 100 ms after finishing S2. The Fourier spectrum of the extracted diastolic heart sound is divided into three modes according to the segmentation boundaries: 150 and 500 Hz using EWT. The frequency distributions of the three modes are 0-150 Hz, 150-500 Hz, and >500 Hz. The spectrums of three modes are obtained through FFT. The first spectral energy between 0 and 150 Hz is denoted as *e*(1). The second spectral energy from 150 to 500 Hz is denoted as *e*(2). The third spectral energy for frequencies higher than 500 Hz is denoted as *e*(3). Every spectral energy is calculated as the square algebraic sum of the amplitude of each frequency value in the frequency band.

### 2.3. Combination of Features of S1 and Diastolic Murmurs

Studies have shown that some heart diseases can also experience weak heart contractions and reduced S1, such as mitral tricuspid regurgitation. There are also some CAD patients with less stenosis of coronary and no obvious weak heart contractions and reduced S1. Therefore, the accuracy of distinguishing CAD from non-CAD by using the parameters of S1 alone is not well.

RETRACTED

It is also feasible to use second diastolic spectral energy *e*(2) alone to identify CAD and non-CAD, but it is also not accurate because diastolic murmurs are not only caused by CAD but also caused by valvular heart disease [4].

Therefore, in order to improve the accuracy in identifying CAD from non-CAD, it is proposed to combine the features of T1, *e*(2), and P3. P3 can be used to identify the diastolic murmurs from CAD and from valvular disease [4]. It is worth noting that when P3 is calculated, the diastolic heart sound spectrum is divided into three different parts: 0~150 Hz, 150~200 Hz, and >200 Hz. P3 is calculated as

(9) $$\begin{array}{c} P_{3}=\frac{E{\left(3\right)}_{f\geq 250\text{ Hz}}}{E{\left(3\right)}_{f<250\text{ Hz}}}, \end{array}$$

where *E*(3) is the third spectral energy.

The performance of this method is evaluated using sensitivity (Se), positive predictivity (Pp), and overall accuracy (Oa), which are defined as

(10) $$\begin{array}{c} \text{Se}=\frac{\text{TP}}{\text{TP}+\text{FN}}\times 100\%,\\ \text{Pp}=\frac{\text{TP}}{\text{TP}+\text{FP}}\times 100\%,\\ \text{Oa}=\frac{\text{TP}}{\text{TP}+\text{FP}+\text{FN}}\times 100\%. \end{array}$$

### 2.4. Description of the Used Database

In this paper, some heart sound signals are from Michigan Heart Sounds and Murmur Database (MHSDB). This database is provided by the University of Michigan Health System. The PCG signals in MHSDB are sampled at 44100 Hz. In order to speed up the signal processing, all the heart sound signals are resampled at 2000 Hz in the pretreatment process. MHSDB includes 23 different clean heart sound recordings from 23 different subjects with a time length of 69 s for each recording. There are about 80 cardiac circles for each recording. The database is intended to teach medical students auscultation and therefore comprises high-quality recordings of very pronounced murmurs [25]. It includes all kinds of heart sounds used in this paper, such as normal heart sound collected at Apex or aortic position, split S1 and S2 collected at apex or aortic position, heart sounds with S4 and S3 collected at apex or aortic position, early, middle, and late diastolic or systolic murmurs collected at apex or aortic position and 3 CAD heart sounds recordings collected at apex position. It is available from https://www.med.umich.edu/lrc/psb/heartsounds/index.htm.

The other part of heart sound signals used in this paper is from Self-Collection Database (SCDB) using MEMS electronic stethoscope as shown in Figure 3 [23]. Its sampling frequency is about 2000 Hz. When the stethoscope's probe shown in Figure 3(b) is placed at the tricuspid valve position of supine human body, the real-time heart sound data collected by the sensor is transmitted to the mobile phone through Bluetooth. The signal to noise ratio (SNR) of heart sound signals collected by MEMS electronic stethoscope is superior to 3200-type of 3 M Littmann stethoscope 8.2 db, which will make the feature extraction of heart sound signals become easier. The measured frequency range is 0~1000 Hz. There are 68 subjects of CAD heart sounds and 50 subjects of healthy heart sounds in SCDB. There are 38 male CAD patients and 30 female CAD patients. Every heart sound recording of CAD has about 40 cardiac circles. Coronary artery occlusion ranges from 30% to 99%.

RETRACTED

## 3. Results and Discussion

### 3.1. Results of Feature Extraction of First Heart Sound

Standard normal S1, S1 of mitral stenosis, S1 split, and S1 of CAD were selected from MHSDB for comparative analysis.  Figure 4 illustrates the spectrum segmentation of different S1 using EWT.

Then, mode decomposition results of different S1 are obtained as shown in Figure 5. They are divided into five modal components. The major components of M1 and T1 in S1 are the two spectral segments containing the selected maximum values. Mode 2 and mode 4 are single frequency components, corresponding to the time domain waveform of T1 and M1.

Figure 6 clearly shows the three-dimensional scatter diagram of IF of M1 and T1 in different S1. The IF of second mode and the fourth mode can form continuous curve after Hilbert Transform and *k*-means clustering analysis. The values of time, frequency, and amplitude corresponding to the IF with the maximum amplitude in M1 and T1 can be easily found. By comparing Figures 6(a)–6(d), it is found that the obvious characteristic that the CAD's S1 differs from other non-CAD's S1 is the value of frequency of M1 and T1's IF significantly reduced. The phenomenon that small amount of regurgitation of the mitral and tricuspid valves was found in most patients with CAD indicated that the mitral and tricuspid valves were not tightly closed in most patients suffering from CAD. Because of weak heart contractions in patients with CAD, resulting in weak mitral and tricuspid valve closure, the IF of M1 and T1 corresponding to mitral and tricuspid valve closure is significantly reduced.

### 3.2. Results of Feature Extraction of Diastolic Murmurs Using EWT

In order to find the difference of diastolic modal spectrum between normal subjects and patients with CAD, a comparative study was carried out.

Figure 7 shows the spectrum segmentation of different diastolic heart sound.  Figure 8 shows the three modes of the two different diastolic heart sounds after the spectrum was divided using EWT.  Figure 9 shows the difference of three modal spectrums between CAD's diastolic heart sounds and normal diastolic heart sounds. It is found that the maximum amplitude of normal diastolic modal spectrum at 150~500 Hz and at 500~1000 Hz is 10^2^ lower than the modal spectral components corresponding to CAD's diastolic heart sounds.

RETRACTED

Then, the spectral energy corresponding to 0~150 Hz modal component was denoted as *e*(1), the spectral energy corresponding to the 150~500 Hz modal component was denoted as *e*(2), and the spectral energy corresponding to the 500~1000 Hz modal component was denoted as *e*(3); Table 1 statistics show *P*_1_ = (*e*(2))/(*e*(1)), *P*_2_ = (*e*(3))/(*e*(1))and the average value of the three modal spectral energy of 6 diastolic heart sounds in normal subject and in patient with CAD. It was found that the diastolic second mode spectral energy *e*(2) significantly increased in patients with CAD. In Table 1, the average value of *e*(2) of CAD is 1.7*e* − 6, while the average value of *e*(2) of normal subject is 2.0*e* − 8. The low-frequency energy (0~150 Hz) of diastolic heart sounds decreased in patients with CAD. The average value of *e*(1) of CAD is 8.6*e* − 4, while this average value of normal subject is 0.0010. In a word, the middle-frequency energy *e*(2) (150~500 Hz) and high-frequency energy *e*(3) (>500 Hz) of CAD's diastolic heart sounds increased significantly. These conclusions are consistent with those of many scholars who have studied the characteristics of diastolic heart sound in CAD [10, 15, 17].

### 3.3. Results of Combination of Features

Table 2 statistics the five characteristic parameters of different heart sounds, which are diastolic second modal spectral energy *e*(2), diastolic third modal spectral energy *e*(3), frequency of M1 and T1 in S1, and P3 which is the ratio of spectral energy greater than 250 Hz to spectral energy less than 250 Hz in the third diastolic mode [4]. The characteristic parameters of each different heart sound are the average relevant value of 40 cardiac cycles. The CAD's heart sounds were mainly collected by MEMS electronic stethoscope on the tricuspid valve position (4 L). Valvular heart disease's heart sounds are mainly from MHSDB.

According to the selection rule, features with the greatest informational entropy in the same attribute, T1, *e*(2), and P3 are selected to compose the feature set and the decision tree classifier is designed based on the statistical data in Table 2.

The decision tree classifier design process takes into account not only the features of CAD itself but also other diseases' features that may interfere with the diagnostic results, such as valvular diseases (mitral stenosis, early and middle diastolic regurgitation murmurs), which lead to an increase in *e*(2) and *e*(3). There are also some diseases that do not have diastolic murmurs but have decreased frequency of T1 and M1, such as elderly themselves with weaken contraction of the heart. Therefore, the design of decision tree needs to combine the features T1, *e*(2), and P3.

RETRACTED

In order to verify the performance of the proposed method in the identification of CAD and non-CAD, comparison experiments were carried out. The methods of empirical mode decomposition (EMD), wavelet analysis, FFT, eigenvector method, an autoregressive (AR) model, and an autoregressive moving average (ARMA) model were chosen for acoustic detection of CAD. The common feature of these methods is that only diastolic analysis of CAD is carried out.

The comparison results show that the proposed algorithm has great advantages over the other method in identification of CAD and non-CAD as shown in Table 3 when considering the other interference heart diseases. There are 50 cases of CAD heart sounds and 50 cases of non-CAD (including normal (20) and valvular disease (30)) heart sounds used in Table 3. The CAD subjects and normal subjects are from SCDB; the other subjects are from MHSDB. The identification results were evaluated using by sensitivity (Se), positive predictivity (Pp), and overall accuracy (Oa) [19] as shown in Table 3. In fact, other methods chosen for comparison experiments mainly studied the difference of diastolic heart sound characteristics between the normal subjects and the CAD subjects and did not consider the interference of valvular diseases on the extraction of diastolic heart sound characteristics of CAD. Therefore, valvular diseases containing diastolic high-frequency murmurs are mostly identified as CAD by other methods, resulting in low Pp and Oa. This paper focuses on how to improve the accuracy of identifying CAD using diastolic heart murmurs. The methods that do not use diastolic murmurs to identify CAD are not the focus of this study.

Table 3 illustrates the superior effectiveness of the proposed method in identification of CAD and non-CAD. The performance of the proposed method can improve the Oa and Pp greatly in identifying CAD and non-CAD when compared with other existing state-of-the-art methods. The proposed method can significantly eliminate the interference of the high-frequency diastolic murmurs from valvular diseases and of the weaken T1 in normal elderly people and greatly improve the accuracy in identification of CAD and non-CAD. With the further accumulation of heart sound data, it is believed that the classification boundary value in the decision tree classifier will become more accurate and perfect, and the data results in Table 3 will also become more accurate and reliable.

RETRACTED

## 4. Conclusion

High-frequency murmurs in diastolic heart sounds are generally believed the typical characteristic of CAD. However, this high-frequency murmurs are usually interfered by the murmurs in valvular disease or high-frequency noise. This paper proposed a method to improve the accuracy in identifying CAD and non-CAD by combining first heart sound characteristic parameter (T1), the second diastolic modal spectral energy *e*(2), and P3. Considering the diastolic murmurs of CAD are easily contaminated by noise and valve sounds, the MEMS electronic stethoscope with high SNR is used to collect heart sounds and wavelet threshold de-noising algorithm is used for denoising firstly. Then, a fixed diastolic window function is selected to extract the diastolic heart sound reflecting maximum coronary blood flow. The EWT algorithm is applied in feature extraction of CAD's S1 and diastolic murmurs. The algorithm for the detection and classification of S1 is described in more detail in Reference [24], and it was applied to extract the characteristic of CAD's S1 in this paper. P3 is mainly used to distinguish diastolic murmurs of CAD and of valvular disease. The algorithm for calculation P3 is proposed in reference [4]. It was found that the significant reduction of T1's frequency in CAD's S1 is a significant characteristic that distinguishes it from other non-CAD's S1. EWT is used to divide the diastolic heart sounds into three modes: 0-150 Hz, 150-500 Hz, and >500 Hz. The modal spectral energy of diastolic heart sounds in CAD subject and in normal subject was calculated, and it was found that the spectral energy of the second mode *e*(2) in CAD patients was significantly higher than that in normal subject. Therefore, the three features—T1, *e*(2), and P3—are combined together to identify CAD and non-CAD. Comparison experiment results show that the performance of proposed method is superior to most existing methods based on diastolic murmurs in identification CAD and non-CAD because the proposed method considered the most interference to the diagnostic rate of CAD when using diastolic murmurs.

## Figures and Tables

**Figure 1:** Trend of mortality of CAD in urban and rural areas from 2002 to 2016.

**Figure 2:** The diagram of the proposed algorithm.

**Figure 3:** The MEMS electronic stethoscope. (a) The installation of the stethoscope. (b) The appearance of the stethoscope.

**Figure 4:** The segmentations of different S1's Fourier spectrum. (a) Normal S1; (b) S1 of mitral stenosis; (c) S1 split; (d) S1 of CAD.

RETRACTED

**Figure 5:** Mode decomposition of different S1. (a) Normal S1; (b) S1 with mitral stenosis; (c) abnormal S1 split; (d) S1 of CAD.

**Figure 6:** Distribution of IF of different S1 after using clustering algorithm. (a) Normal S1; (b) S1 with mitral stenosis; (c) abnormal S1 split; (d) S1 of CAD.

**Figure 7:** Diastolic spectrum segmentation. (a) CAD's diastolic spectrum segmentation; (b) normal diastolic spectrum segmentation.

**Figure 8:** Modal decomposition of two different diastolic heart sounds. (a) CAD's diastolic heart sounds; (b) normal diastolic heart sounds.

**Figure 9:** Spectrum of diastolic modes. (a) Spectrum of CAD's diastolic modes; (b) spectrum of normal diastolic modes.

**Algorithm 1:** .

**Table 1:** Comparison of characteristic values between CAD and normal subject.

CAD						Normal subject				
No.	*e*(1) V^2^·s	*e*(2) V^2^·s	*e*(3) V^2^·s	P1	P2	*e*(1) V^2^·s	*e*(2) V^2^·s	*e*(3) V^2^·s	P1	P2
1	0.0015	2.8*e* − 6	1.7*e* − 7	0.0018	1.1*e* − 4	3.4*e* − 4	2.2*e* − 8	1.8*e* − 10	6.4*e* − 5	5.4*e* − 7
2	3.8*e* − 4	1.1*e* − 6	8.9*e* − 8	0.0028	2.3*e* − 4	3.8*e* − 4	3.4*e* − 8	3.4*e* − 10	8.8*e* − 5	8.8*e* − 7
3	7.7*e* − 4	1.9*e* − 6	1.5*e* − 7	0.0025	2.0*e* − 4	9.8*e* − 4	1.6*e* − 8	6.9*e* − 11	1.6*e* − 5	7.0*e* − 8
4	0.0015	1.9*e* − 6	2.4*e* − 7	0.0013	1.6*e* − 4	0.0014	2.1*e* − 8	1.8*e* − 10	1.5*e* − 5	1.3*e* − 7
5	6.2*e* − 4	1.5*e* − 6	1.0*e* − 7	0.0024	1.7*e* − 4	0.0017	1.0*e* − 8	7.8*e* − 11	6.0*e* − 6	4.5*e* − 8
6	4.0*e* − 4	1.1*e* − 6	8.4*e* − 8	0.0029	2.1*e* − 4	0.0013	1.6*e* − 8	1.7*e* − 10	1.2*e* − 5	1.3*e* − 7
*μ*	8.6*e* − 4	1.7*e* − 6	1.4*e* − 7	0.0023	1.8*e* − 4	0.0010	2.0*e* − 8	1.7*e* − 10	3.4*e* − 5	3.0*e* − 7
*δ*	2.2*e* − 7	3*e* − 13	3*e* − 15	3.1*e* − 7	1.5*e* − 9	2.6*e* − 7	5.6*e* − 17	8.0*e* − 21	9.6*e* − 10	9.5*e* − 14

**Table 2:** The relationship between heart sound characteristics and CAD or non-CAD.

No.	Source	Recordings	*e*(2) (V2·s)	*e*(3) (V2·s)	M1 (Hz)	T1 (Hz)	P3	Is it CAD?	Note
1	SCDB	40 cardiac cycles	4.80*e* − 6	3.49*e* − 7	28	6	19.3	Yes	50% coronary blockage
2	SCDB	40 cardiac cycles	5.23*e* − 6	3.56*e* − 7	19	4	25.14	Yes	60% coronary blockage
3	MHSDB	40 cardiac cycles	2.2*e* − 8	1.8*e* − 10	39	10	16.19	No	Normal
4	SCDB	40 cardiac cycles	2.43*e* − 5	1.45*e* − 6	22	8	10.17	Yes	90% coronary blockage
5	SCDB	40 cardiac cycles	3.58*e* − 5	1.90*e* − 6	27	6	62.46	Yes	Multiple coronary blockages
6	SCDB	40 cardiac cycles	1.29*e* − 6	5.93*e* − 8	23	4	8.96	Yes	50% coronary blockage
7	SCDB	40 cardiac cycles	1.58*e* − 5	6.33*e* − 7	46	6	9.98	Yes	90% coronary blockage
8	MHSDB	40 cardiac cycles	2.23*e* − 8	9.89*e* − 8	47	22	7.38	No	Mitral stenosis
9	MHSDB	40 cardiac cycles	0	0	51	13	0.92	No	Late diastolic valve murmurs
10	SCDB	40 cardiac cycles	3.42*e* − 5	1.77*e* − 6	18	4	48.16	Yes	Multiple coronary blockages
11	MHSDB	40 cardiac cycles	3.66*e* − 7	4.63*e* − 8	21	7	0.86	No	Early and late valve diastolic murmurs
12	SCDB	40 cardiac cycles	1.45*e* − 7	5.76*e* − 9	60	21	1.35	No	Normal

RETRACTED

**Table 3:** Comparison of the performance of different method in identification of CAD and non-CAD.

Different methods	Total subjects	TP	FN	FP	Se (%)	Pp (%)	Oa (%)
HHT	100	50	10	31	83.3	61.7	54.9
Wavelet analysis	100	48	12	28	80	63.1	54.5
Eigenvector method	100	51	9	26	85	66.2	59.3
AR model	100	49	11	33	81.2	59.8	52.7
ARMA	100	47	13	35	78.3	57.3	49.5
Proposed method	100	55	5	4	91.2	93.2	85.9

## Data Availability

Data sharing is not applicable to this article as no datasets were generated or analyzed during the current study.
